The article "Assessment of Seasonal Radon Concentration in Dwellings and Soils in Selected Areas in Ga East, Greater Accra Region of Ghana" was published in 2022. Journal: J Environ Public Health.

# Assessment of Seasonal Radon Concentration in Dwellings and Soils in Selected Areas in Ga East, Greater Accra Region of Ghana

**DOI:** 10.1155/2022/6600919

**Published:** 2022-08-24

**Authors:** R. Kpordzro, J. K. Gbadago, A. B. Andam, O. K. Adukpo, F. Otoo, I. Opoku-Ntim, M. Abubakar, E. Amoatey

**Affiliations:** ^1^Radiation Protection Institute, Ghana Atomic Energy Commission, P. O. Box LG 80, Legon, Accra, Ghana; ^2^School of Nuclear and Allied Sciences, University of Ghana, P. O. Box AEI Atomic Campus, Accra, Ghana; ^3^National Nuclear and Research Institute Atomic Energy Commission, P. O. Box LG 80, Legon, Accra, Ghana

## Abstract

Seasonal radon levels have been studied in dwellings and soils in selected areas in Ga East, Greater Accra Region of Ghana using LR-115-type II (SSNTDs). This study was conducted to determine the seasonal correlation between soil and dwelling radon concentrations. Detectors were exposed from January to March and April to June, for dry and wet seasons, respectively. Overall, indoor radon was 133.4 ± 6.7 Bqm^−3^ and 72.1 ± 3.6 Bqm ^−3^ for wet and dry seasons. The estimated annual effective dose to the lung received by the occupants at Paraku Estate, Dome, and Kwabenya was 6.9 ± 0.4, 7.2 ± 0.5, and 9.8 ± 0.8 mSvy^−1^ for the wet season and 3.8 ± 0.2, 4.3 ± 0.2, and 4.6 ± 0.3 mSvy^−1^ for the dry season. On average, the soil radon concentration was found to be 0.96 ± 0.07 kBqm^−3^ and 2.24 ± 0.01 kBqm^−3^ for wet and dry seasons. To determine the correlation between soil and dwelling radon, a positive Pearson correlation coefficient value R = (0.74) and R = (0.66) was obtained representing the dry and wet seasons. To test the statistical significance between soil and dwelling radon, *P* < 0.05 was obtained, indicating a statically significant relationship between the two.

## 1. Introduction

Radon gas is from the natural radioactive decay of uranium, thoron, and actium originally from underground bedrocks and soils. These natural radionuclides produce the three natural isotopes of radon, namely, Radon^222^, Radon^220^, and Radon^219^. According to UNSCEAR 2000, the contribution of radiation dose from Radon^220^ and Radon^219^ is generally insignificant because of their short half-life [1]. The radioisotope Radon^222^ with a half-life of 3.8 days decays into a short-lived series of progeny which emits high-energy alpha particles, and two of these are polonium-218 and polonium-214. Because alpha particles are electrostatic, they can adhere to particulates in the environment and become radioactive pollutants in the atmosphere [2]. This is a major source of concern since it has significant implications for public health and the environment. There are several air pollutants, including lead from radon progenies, according to the World Health Organization. Long- and short-term exposure to this suspended pollution can cause respiratory and cardiovascular problems, as well as neuropsychiatric difficulties, eye irritation, skin diseases, autism, and long-term chronic diseases including cancer. Several reports have identified the direct link between exposure to radon and the increasing rate of morbidity and mortality [3–8].

The article "Assessment of Seasonal Radon Concentration in Dwellings and Soils in Selected Areas in Ga East, Greater Accra Region of Ghana" was published in 2022. Journal: J Environ Public Health.

Radon gas is found everywhere, and their concentrations are low outdoors but can build up indoors, especially in homes, where most exposure of the general population occurs. Studies in Europe, North America, and China have confirmed that a low concentration of radon such as those commonly found in residential settings also poses a health risk and contributes to the occurrences of lung cancers worldwide increased by about 16% per 100 Bqm^−3^ in a long-term average radon concentration [9,10]. The average outdoor radon level varies from 5 Bqm^−3^ to 15 Bqm^−3^. However, levels are higher in indoor environments, especially areas with minimal ventilation; radon levels can vary substantially from 10 Bqm^−3^ to more than 10000 Bqm^−3^. In 2010, ICRP published a comprehensive review of the science relating lung cancer to radon exposure (ICRP Publication 115 Lung Cancer Risk from Radon and Progeny and Statement on Radon). Based on scientific evidence at the time, the recommended maximum reference level, a key figure driving public health policy for indoor radon, was reduced to 300 Bqm^−3^ [11]. The WHO's recommendations are the same: a national reference level of 100 Bqm^−3^ is suggested, and if this is not possible, the chosen level should not exceed 300 Bqm^−3^. In line with these standards, countries such as Denmark, Belgium, Canada, Brazil, France, Estonia, and others have come up with guidelines levels in dwellings similar to the maximum levels recommended by WHO and ICRP, except for the United States of America whose reference level is 148 Bqm^−3^ [12].

The World Health Organization, the United States Environmental Protection Agency, and other private entities have developed mitigation measures that can be used to reduce radon levels when they exceed WHO-recommended upper limits and country-specific reference levels. Some of them prevent radon from entering the structure, while others reduce the concentration of radon once it has. Soil suction, perforated pipe, drain tile or sump-hole suction, submembrane suction, sealing foundation cracks and openings, home pressurization or use of air-to-air heat exchangers, and natural ventilation, which is a temporary solution because it can affect air conditioning and home security [13–16].

The article "Assessment of Seasonal Radon Concentration in Dwellings and Soils in Selected Areas in Ga East, Greater Accra Region of Ghana" was published in 2022. Journal: J Environ Public Health.

Much has not been done in Ghana in terms of radon assessment, and there are currently no national guideline levels. The results of studies on radon gas in dwellings and the soil were higher than the WHO and ICRP reference levels [17–21]. Most studies on radon concentrations, on the other hand, have only focused on radon in soil and radon in dwellings separately. To account for the high levels of dwelling radon gas in these areas, the current study seeks to conduct a systematic assessment of soil and dwelling radon in the same study area. Radon gas in the soil is of special relevance because it is the population's primary source of natural radiation exposure. Within the district, radon studies have only looked at dwelling radon, not soil radon gas measurement [17, 18]. The current study aimed to conduct a comprehensive assessment of soil and dwelling radon to account for the high levels of dwelling radon gas in the district.

## 2. Materials and Methods

This study was not approved by any ethical clearance committees, since the Nuclear Regulatory Authority in the country does not mandatorily apply to this type of environmental study.

### 2.1. Description of the Study Area

Ghana has sixteen regions; the research area is in Ghana's Greater Accra region, within the Ga East Municipal Assembly (GEMA). It is bounded to the north and south by the Akwapim-Togo ranges and the Ga district. Akwapim-Togo ranges are identified as one of the areas in the country with fault lines, which run through Ga east Accra. The area is predominantly underlined by middle to late Proterozoic rock units also known as Dahomevan, Togo, Buem, and Voltain belt [22]. Ghana has a tropical climate that is heavily impacted by the West African monsoon winds. The weather is generally warm with seasons and elevations masking temperature variations. The northern half of the country has only one rainy season, whereas the southern part has two: a major season from April to July and a minor season from September to November. Several climate models have confirmed that the rate of increase in temperature has generally been more rapid in the northern parts than the southern parts. Due to the African monsoon, the dry season in Ghana is referred to as the winter and the rainy season is referred to as summer [23] As indicated in Figure 1, the study location and the sampling sites are Dome, Paraku estate, and Kwabenya all of which are located in Ghana's southern region.

### 2.2. Experimental Design

Seasonal radon assessment was carried out in this study for both indoor and soil radon. LR 115 type II Solid State Nuclear Track Detectors (SSNTDs) obtained from Kodak Pathé, France, were used for the radon measurement. During the sampling selections, a building with the same construction materials as sandcrete buildings with an average of two windows and ground floor was chosen. However, the flooring materials of the dwelling in the different areas differ from each other. Tiled, cemented, and raw concrete floors were chosen for Paraku Estate, Dome, and Kwabenya. This was considered to assess the entry rate of radon into the dwellings through these roots.

The article "Assessment of Seasonal Radon Concentration in Dwellings and Soils in Selected Areas in Ga East, Greater Accra Region of Ghana" was published in 2022. Journal: J Environ Public Health.

Two techniques of measuring radon were employed for this study. The passive radon monitoring technique was used for the indoor radon measurement, and the in situ radon technique was used for the soil radon measurement. All the procedures used for both indoor and soil measurement in this current study were standard procedures that have been used in Ghana for several radon studies including intercomparison exercises [17, 18, 20, 21, 24–26].

- The indoor radon passive assessment was from January to March 2020, representing the dry season, and then April to June 2020 for the rainy season. Detector deployment was done in individual bedrooms. Twenty (20) dwellings in each of the locations were selected to ensure quality control, duplicate measurement was done for both the dry and the wet seasons, and a total of 240 detectors were used.
- In situ soil radon measurement was done in the immediate environments where indoor radon was carried out. Thirty (30) radon detectors were exposed for 14 days for two cycles in each season. A total of one hundred and twenty (120) detectors were used.

### 2.3. Indoor Radon Measurements

The LR 115 Types II Solid-State Nuclear Track Detectors (SSNTD) were cut into rectangular sizes (2 cm × 3 cm). The detectors were kept in a specially designed envelope to hold the detectors in place. With the aid of masking tape, the envelopes with their detectors were fixed on the wall, about 2 m in the varied flooring material dwellings. This was done to be able to quantify the entry rate of radon diffusion through the different floor materials in the dwellings. In each dweller's bedroom, the detectors were placed away from windows and doors. Approximately two-third parts of the detectors were exposed to capture the radon decay products in the room. The one-third portion of the detectors inside the envelope which was not covered was used to compare the intrinsic factory reading. The detector exposure was done for three months in each of the seasons.

### 2.4. Etching and Counting of Tracks

After 3 months of exposure for every season, the detectors were then subjected to a chemical etching process in a 2.5 N sodium hydroxide (NaOH) solution at a constant temperature of 60 ± 1°C for 1 hr 30 min. Afterwards, the detectors were rinsed under running tap water and then in distilled water. They were air-dried for 24 hours and then counted. A commercial scanner (Epson Perfection V600) and Image J digital image processing software were used for the image processing and counting of alpha tracks registered by the detectors [24, 27].

The article "Assessment of Seasonal Radon Concentration in Dwellings and Soils in Selected Areas in Ga East, Greater Accra Region of Ghana" was published in 2022. Journal: J Environ Public Health.

### 2.5. Soil Radon Measurement

In situ soil radon gas assessment was performed using the closed tube method, as indicated in Figure 2. The tubes were made of polyvinyl chloride plastic with a length of 25 cm; this was buried in a dug hole at a depth of about 75 cm. The detectors were cut into sizes of 2 cm × 2 cm and were attached to the bottom of a wooden stopper, fitted into the tube, and placed in the dug hole. The distance between the detector and the soil surfaces caused a negligible contribution of thoron from reaching the detectors because it decays before reaching the effective surface of the detector. The distribution of Rn^220^ atoms exhaled from the soil surface decreases exponentially with distance inside the tube. It is known that the diffusion length of Rn^220^ atoms is approximately 2-3 cm in the air compared to the diffusion length of Rn^222^ atoms with approximately 239 cm. Therefore, more than 90% of the Rn^222^ atoms from the soil could reach the detector [28]. The holes were then covered first with an aluminum sheet and then with sand to assume a normal environmental condition. The soil environment in the dry season was dry and less humid; it was moist and humid in the wet season. After exposure, the detectors were removed from the wooden stoppers and sent to the laboratory. The alpha tracks registered by the detectors were prepared, etched, scanned, and counted using the same methodology as described in section 2.4 [21, 29].

### 2.6. Data Analysis

#### 2.6.1. Track Density

The number of tracks per unit surface is measured in a direction perpendicular to the direction in which the tracks are read.

(1) $$\begin{array}{c} \text{Track Density}\left(\rho \right)=\frac{\text{Average number of counts}}{\text{Area of electrode}}. \end{array}$$

The concentration of indoor radon gas (Bqm^−3^) and soil radon (kBqm^−3^)

(2) $$\begin{array}{c} \text{Concentration CRn}\left(Bqm-3\right)=\frac{\rho -\rho B}{Ε\times T},\\ \text{Concentration}\left(kBqm^{-3}\right)=\frac{\rho -\rho B}{Ε\times T*}, \end{array}$$

where *ε* is the calibration factor of LR-115, Type II detector = 3.96 (Tracks.m^3^/cm^2^ kBq.h). T is the exposure time = 90 days for indoor passive monitoring. *T∗* is the exposure time = 14 days for in situ soil radon monitoring. *ρB* is the background track density = average count on the unexposed part of the detectors, and *ρ* is the measured surface density of tracks (tracks/cm^2^).

The article "Assessment of Seasonal Radon Concentration in Dwellings and Soils in Selected Areas in Ga East, Greater Accra Region of Ghana" was published in 2022. Journal: J Environ Public Health.

#### 2.6.2. Annual Effective Dose (mSvyr^−1^)

The annual effective dose (*E*) of exposure to indoor radon gas in dwellings was calculated using the equation proposed by UNSCEAR 2000 [1].

(3) $$\begin{array}{c} E=C_{Rn}\times O_{f}\times D_{f}\times I_{f}\times T_{y}, \end{array}$$

where *C*_*Rn*:_ is the arithmetic mean of indoor radon concentration in dwellings, *O*_f_ is the indoor occupancy factor of 0.8, and *D*_*f*_ is the dose conversion factor of (9 × 10^−6^ mSvh^−1^ per Bqm^−3^). *I*_f_ is the indoor radon equilibrium factor (0.4). *T*_y_ is time in hours in a year (24 h × 365 days = 8,760 hrs·yr^−1^)

#### 2.6.3. Annual Effective Dose to the Lungs (*E*_L_) (mSvyr^−1^)

The resultant annual effective dose to the lungs (*E*_L_) from exposure to indoor radon gas received by the occupants was estimated using

(4) $$\begin{array}{c} EEL=EE\times WR\times WT, \end{array}$$

where *E* is the annual effective dose of exposure to indoor radon gas (mSvyr^−1^.). *W*_R_ is the radiation weighting factor value of (20) for alpha particles, and *W*_T_ is the tissue weighting factor of (0.12) for the lung [30].

## 3. Results

### 3.1. Seasonal Indoor Radon Concentrations Relative to the Flooring Material of Dwellings

Seasonal radon measurement was conducted in sixty (60) dwellings with different flooring materials at different locations. All the other factors considered for the investigations were the same.  Figure 3(a) and 3(b) are a frequency distribution, describing radon concentration reports in all sixty (60) dwellings in the wet and dry seasons. The graph looked log normal for both seasons. The highest and lowest frequency reported for the dry season was 80 and 130 Bqm^−3^, whereas the rainy season was 80 and 340°Bqm^−3^.  Table 1 gives a summary of minimum and maximum arithmetic mean of indoor radon concentration, and their corresponding annual effective dose to the lungs in the study areas. The arithmetic means recorded for Paraku Estate, Dome, and Kwabena in the wet season were 115.9 ± 5.8, 119.3 ± 5.9, and 165.1 ± 8.3 Bqm^−3^, respectively. The dry season also recorded 66.1 ± 3.7, 73.1 ± 3.3, and 77.1 ± 3.8 Bqm^−3^. These values were then estimated for the annual effective dose to the lungs to obtain 6.9 ± 0.4, 7.2 ± 0.5, and 9.8 ± 0.8 mSvy^−1^ for wet and 3.8 ± 0.2, 4.3 ± 0.2, and 4.6 ± 0.3 mSvy^−1^ in the dry seasons for Paraku Estate, Dome, and Kwabenya.

### 3.2. Indoor Radon Compared with Soil Radon in Both Seasons

Soil radon measurement was carried out in an immediate environment where indoor radon was measured. Thirty sites were located and dug for soil radon. However, twenty-three detectors were retrieved, and the analysis was based on the detectors that were retrieved. As indicated in Figures 4(a) and 4(b), the soil radon concentrations in the dry seasons are higher than that of their corresponding indoor concentration in the same season; this is also the same for soil radon concentrations obtained in the rainy season.  Table 2 describes the radon concentration obtained in the first and second count of the tracks which was registered by the detectors, with their average concentrations and standard deviations for both the wet and dry seasons. Detector location (DL1) had the highest counts, with an average of 1.79 ± 0.27 kBqm^−3^, and the lowest count was reported to be found in (DL7) with an average of 0.09 ± 0.01 kBqm^−3^ for the rainy season. On the other hand, the dry season ranged from 0.19 ± 0.01 to 3.39 ± 0.50 kBqm^−3^ funds in detector location (DL21) and (DL19). The arithmetic mean for the wet and dry seasons was 0.96 ± 0.07 kBqm^−3^ and 2.24 ± 0.01 kBqm^−3^, respectively.

The article "Assessment of Seasonal Radon Concentration in Dwellings and Soils in Selected Areas in Ga East, Greater Accra Region of Ghana" was published in 2022. Journal: J Environ Public Health.

### 3.3. Correlation between Soil and Indoor Radon

Indoor and soil radon data in the study locations have been summarized in Figures 5(a) and 5(b); a positive Pearson's correlation coefficient R = (0.740) and (0.659) for dry and wet seasons were observed. These values were translated indirectly into a *T*–a value of (5.052806) and (4.021314). To test the statistical significance between soil and indoor radon in the study area, a *P* value (<0.05) was obtained in both seasons.

### 3.4. Comparison of Indoor Radon Levels in Ghana and Other Countries

The indoor radon concentration obtained in the current study was compared with works done in Ghana and other countries in Table 3. Considering radon exposure and its health risk, the World Health Organization came up with a comprehensive decision on the radon reference level of 100 Bqm^−3^ and not exceeding 300 Bqm^−3^ for indoor radon. Several countries have established country-specific guidelines in line with this recommendation. Currently, the compilation of radon data is ongoing in Ghana [38]. Indoor radon concentrations recorded in Dome [17] in the previous study were 466.9 Bqm^−3^ higher than the exceeding limit by [16]. The concentration obtained in [18] was 121 Bqm^−3^ closer to the values obtained in this current study. Except for Refs. 17, 20, the rest of the data obtained were within the WHO upper limit of 300 Bqm^−3^.

## 4. Discussion

It is critical to study seasonal indoor and soil radon systematically because soil radon is one of the population's primary sources of natural radiation exposure. Increased radon levels play a major role in the occurrence of a variety of diseases, including cancers, and this can also be a result of rapid climate changes, which sometimes cause major harm to public health and properties. During the rainy season, windows and doors are closed, which can result in the accumulation of indoor radon gas pollutants in dwellings. However, in the dry season, windows are frequently opened for some of the indoor gas to escape from dwellings, causing a reduction in radon levels during the dry season. Variations in reported seasonal indoor radon concentrations as indicated in Section 3.1 can be observed. The arithmetic means of indoor radon concentration obtained in the rainy season is higher compared with its corresponding concentration in the dry season. This can be attributed to the reasons mentioned above. This report is in agreement with studies conducted by [39–41].

The article "Assessment of Seasonal Radon Concentration in Dwellings and Soils in Selected Areas in Ga East, Greater Accra Region of Ghana" was published in 2022. Journal: J Environ Public Health.

The frequency distribution for each season was log-normal; the reason for the lack of a normal distribution can be attributed to the different flooring materials, which allowed radon to enter the dwelling at different rates through the foundation walls of the buildings. The mean values obtained in Paraku Estate are lower than the mean values obtained in Dome and Kwabenya. This was because the tiled floor material used in Paraku Estate dwellings delayed radon diffusion into the dwellings, whereas the cemented and exposed concrete floors at Dome and Kwabenya contributed to the rapid diffusion of radon into the dwellings.

The frequency distribution is positively skewed, indicating that majority of the data points are low. Concentrations of more than 100 Bqm^−3^ were found in 20% of the total dwellings monitored [11, 16]. The overall annual indoor radon concentration in the study area was found to be 102.7 ± 5.1 Bqm^−3^, a little above the reference level mentioned in Refs [11, 16], but within the recommended maximum limit of 300 Bqm^−3^. The estimated annual effective dose to the lung received by the occupants in the study area was 6.1 mSvy^−1^. This value is lower than the maximum limit equivalent to 17 mSvy^−1^, recommended by ICRP in 2010.

In the comparison analysis between soil and indoor radon gas, reported in Section 3.2 and Figures 4(a) and 4(b), the average soil radon concentrations in almost all the sites that were dug in both seasons showed a significant variation between the soil radon and indoor radon. The soil radon in both seasons was higher than the corresponding indoor radon. This can be attributed to the fact that within the soil, there is a relatively higher amount of radium-226 which produces more radon-222. However, other factors could affect the diffusion of radon from the soil through the foundation walls into the dwellings, particularly the nature of the flooring material and other meteorological factors. These could account for the low radon in dwellings as compared to the radon levels in the soil. This report is not different from the results in [37, 42].

The article "Assessment of Seasonal Radon Concentration in Dwellings and Soils in Selected Areas in Ga East, Greater Accra Region of Ghana" was published in 2022. Journal: J Environ Public Health.

The set of data was analyzed to investigate the seasonal variability of soil-gas radon concentration in the study area, which has similar geological conditions and climate. The results revealed significant variations in the soil radon concentrations measured in the dry and rainy seasons.  Table 2 reports the results of soil radon concentration values obtained in the first and second counts with their average radon concentrations and standard deviations in the different seasons. Soil radon in the dry season was higher than that in the rainy season. This was largely attributed to the fact that there were water-saturation and moisture-retention characteristics of the dug areas of the soil during the rainy season and less water and moisture during the dry season. Radon tended to be confined underground by the water-saturated surface soil, which had much-reduced radon gas permeability, while during the dry seasons, it exhaled faster as the soil became drier and more permeable. These results are not different from the results obtained from studies conducted by Refs [41, 43–45].

Soil radon levels were correlated with indoor radon. This is reported in section 3.3, Figures 5(a), and 5(b). The results show a positive correlation between indoor and soil radon in both seasons. The values were then tested and converted into a *P* value (0.05), indicating that there was a significant relationship between soil radon and indoor radon.

It is important that the indoor radon assessment conducted in the current study be compared with previous studies in Ghana and other parts of the world. Indoor radon concentrations obtained from [17] were higher than the concentrations obtained in the current study, but closer to those of Ref. [18]. This could generally be attributed to the meteorological conditions in the areas since radon concentration can change with time. The results obtained in Nigeria, Hungary, and Saudi Arabia were lower than the values obtained in the current study and below the recommended reference level by WHO. Turkey, Kenya, and Pakistan recorded concentration values higher than the values obtained in the current study.

## 5. Conclusion

The study demonstrated seasonal variations in dwelling and soil radon in some selected areas in Ga East, Greater Accra Region of Ghana. This was motivated by the fact that no systematic assessments of soil and dwelling radon have been conducted at the study locations to account for the high radon levels reported in the area [17].

The article "Assessment of Seasonal Radon Concentration in Dwellings and Soils in Selected Areas in Ga East, Greater Accra Region of Ghana" was published in 2022. Journal: J Environ Public Health.

From the findings, the study did not demonstrate a high risk of radon concentration in Ga East, Accra dwellings as reported in the results obtained in the previous studies. However, it is recommended that comprehensive monitoring activities should be implemented to better describe this environmental pollutant. The mean indoor radon concentration in the area did not exceed the upper limit recommended by the World Health Organization and the international commission on radiological protection. Though the majority of the data points were low, about 20% of the results were above 100 Bqm^−3^. Therefore, it is recommended that continuous education is needed to improve human behavior, focusing on the importance of natural ventilation.

The study was carried out on dwelling construction with different flooring materials to establish the type that will aid in the fast entry rate of radon diffusion in dwellings at various locations. The results showed a significant difference in the dwelling concentration in the various locations. The values obtained in Kwabenya and Dome compared to those of Paraku Estate were higher; therefore, the inhabitants were advised to use tiles as flooring material to seal all available entry points of radon diffusion into the dwellings.

The soil radon concentrations obtained in both seasons were higher than their corresponding indoor radon concentrations. However, the correlation between soil and dwelling radon gave a positive Pearson correlation in both seasons, indicating a statically significant relationship between the two. This report on soil radon gas measurement is useful in assessing dwellings having high radon levels. These data obtained will be added to the existing data to come up with a radon reference level for Ghana.

## Figures and Tables

**Figure 1:** Map of sampling area.

**Figure 2:** Set up of soil radon sampling.

**Figure 3:** Frequency distribution of indoor radon concentration in dry (a) and wet (b) seasons.

**Figure 4:** Comparison of soil and indoor radon concentrations in the wet (a) and dry (b) seasons.

**Figure 5:** (a, b) Correlation analysis between soil vs. indoor radon in dry and wet seasons.

**Table 1:** Radon concentrations and corresponding mean and annual effective dose to the lungs in the study areas.

Location	^222^Rn con. Wet season (Bqm^−3^)		Mean (Bqm^−3^)	Annual effective dose (mSvy^−1^)	Annual effective dose to lungs (mSvy^−1^)	222Rn con. Dry season (Bqm−3)		Mean (Bqm−3)	Annual effective dose (mSvy^−1^)	Annual effective dose to lungs (mSvy−1)
	Min	Max				Min	Max			
Kwabenya	87.4 ± 4.4	334.1 ± 16.7	165.1 ± 8.3	4.1 ± 4.4	9.8 ± 0.8	42.8 ± 2.1	124.1 ± 6.2	77.1 ± 3.8	1.9 ± 1.3	4.6 ± 0.2
Paraku Estate	53.4 ± 2.7	229.2 ± 11.5	115.9 ± 5.8	2.9 ± 2.9	6.9 ± 0.4	51.3 ± 3.5	117.2 ± 5.9	66.1 ± 3.7	1.8 ± 0.9	3.8 ± 0.2
Dome	75.7 ± 3.8	177.4 ± 8.9	119.3 ± 5.9	3.0 ± 2.2	47.6 ± 2.4	184.6 ± 3.4	73.1 ± 0.3.3	1.6 ± 0.6	4.3 ± 0.2	

The article "Assessment of Seasonal Radon Concentration in Dwellings and Soils in Selected Areas in Ga East, Greater Accra Region of Ghana" was published in 2022. Journal: J Environ Public Health.

**Table 2:** Soil radon concentration in 1^st^ and 2^nd^ count with their standard deviations in both seasons.

Detector locations (DL)	1^st^ count	2^nd^ counts	Average	1^st^ count	2^nd^ count	Average
	Wet season (kBqm^−3^)			Dry season (kBqm^−3^)		
DL 1	1.782 ± 0.27	1.798 ± 0.26	1.790 ± 0.27	0.450 ± 0.02	0.456 ± 0.01	0.456 ± 0.002
DL 2	0.783 ± 0.01	0.777 ± 0.02	0.780 ± 0.02	1.956 ± 0.25	1.947 ± 0.24	1.951 ± 0.26
DL 3	0.841 ± 0.09	0.859 ± 0.08	0.850 ± 0.08	0.252 ± 0.01	0.268 ± 0.02	0.260 ± 0.02
DL 4	0.172 ± 0.02	0.168 ± 0.01	0.170 ± 0.01	0.953 ± 0.10	0.967 ± 0.09	0.960 ± 0.09
DL 5	0.913 ± 0.07	0.927 ± 0.08	0.920 ± 0.08	1.406 ± 0.20	1.394 ± 0.18	1.400 ± 0.19
DL 6	0.984 ± 0.09	0.976 ± 0.08	0.980 ± 0.10	1.540 ± 0.22	1.530 ± 0.21	1.535 ± 0.23
DL 7	0.087 ± 0.01	0.101 ± 0.02	0.094 ± 0.01	0.832 ± 0.07	0.838 ± 0.06	0.835 ± 0 .05
DL 8	0.150 ± 0.02	0.168 ± 0.01	0.159 ± 0.02	0.861 ± 0.08	0.879 ± 0.07	0.870 ± 0.06
DL 9	0.915 ± 0.09	0.905 ± 0.08	0.910 ± 0.09	1.484 ± 0.20	1.476 ± 0.17	1.480 ± 0.18
DL 10	1.399 ± 0.14	1.381 ± 0.13	1.390 ± 0.14	0.951 ± 0.09	0.949 ± 0.08	0.950 ± 0.07
DL 11	0.990 ± 0.09	0.988 ± 0.08	0.989 ± 0.09	0.537 ± 0.03	0.543 ± 0.04	0.540 ± 0.02
DL 12	0.667 ± 0.05	0.673 ± 0.06	0.970 ± 0.08	1.370 ± 0.21	1.364 ± 0.20	1.367 ± 0.19
DL 13	0.135 ± 0.01	0.127 ± 0.01	0.131 ± 0.01	0.683 ± 0.05	0.697 ± 0.04	0.690 ± 0.02
DL 14	0.478 ± 0.02	0.462 ± 0.01	0.470 ± 0.02	0.562 ± 0.03	0.550 ± 0.02	0.556 ± 0.04
DL 15	1.010 ± 0.10	1.020 ± 0.11	1.015 ± 0.12	0.994 ± 0.10	0.976 ± 0.11	0.985 ± 0.09
DL 16	0.524 ± 0.03	0.536 ± 0.02	0.530 ± 0.03	1.082 ± 0.16	1.078 ± 0.14	1.080 ± 0.12
DL 17	0.200 ± 0.01	0.180 ± 0.01	0.190 ± 0.01	0.975 ± 0.09	0.991 ± 0.08	0.983 ± 0.06
DL 18	0.913 ± 0.08	0.927 ± 0.09	0.920 ± 0.09	2.034 ± 0.31	2.025 ± 0.29	2.030 ± 0.27
DL 19	0.195 ± 0.01	0.199 ± 0.01	0.197 ± 0.02	3.389 ± 0.51	3.391 ± 0.53	3.390 ± 0.50
DL 20	0.186 ± 0.01	0.186 ± 0.01	0.185 ± 0.02	0.965 ± 0.10	0.975 ± 0.13	0.970 ± 0.14
DL 21	0.129 ± 0.01	0.143 ± 0.01	0.136 ± 0.02	0.197 ± 0.01	0.183 ± 0.02	0.190 ± 0.01
DL 22	0.154 ± 0.01	0.146 ± 0.01	0.150 ± 0.03	2.336 ± 0.35	2.346 ± 0.33	2.341 ± 0.32
DL 23	0.609 ± 0.04	0.591 ± 0.03	0.600 ± 0.04	1.846 ± 0.28	1.834 ± 0.27	1.840 ± 0.26

**Table 3:** Comparison of indoor radon levels in current study with studies in Ghana and other countries.

Country	Areas monitored	Average concentration (Bqm^−3^)	Range (Bqm^−3^)	Ref
Ghana	Dome	119.6	75.7-177.4	—
Ghana	Kwabenya	165.1	87.4-334.1	—
Ghana	Paraku Estate	155.9	53.4-229.2	—
Ghana	Dome	466.9	278.1-740.1	[17]
Ghana	Dome	121	5-325	[18]
Ghana	Kassenna—Nakana	132.7	35.3-244.2	[19]
Ghana	South eastern	518.7	169.3-2047.7	[20]
France	Brittany	155	—	[31]
Nigeria	South western	39	5-255	[32]
Turkey	Giresun	130	52-360	[33]
Kenya	—	170.3	30.2-315.4	[34]
Hungary	—	58	10-5800	[35]
Pakistan	Hazara	128	41-254	[36]
Saudi Arabia	Jeddah	36	21-52	[37]

The article "Assessment of Seasonal Radon Concentration in Dwellings and Soils in Selected Areas in Ga East, Greater Accra Region of Ghana" was published in 2022. Journal: J Environ Public Health.

## Data Availability

Data supporting the finding of this study are included in the manuscript in the form of tables and figures cited in the main text.

## References

[1] UNSCEAR (2000). *Sources, Effect, and Risk of Ionizing Radiation. United Nations Scientific Committee on the Effects of Atomic Radiation*.

[2] Levels O. (2016). Studies of radon in ireland: outdoor levels, detector intercomparison and school remediation methods.

[3] López-Abente G., Núñez O., Fernández-Navarro P. (2018). Residential radon and cancer mortality in Galicia, Spain. *Science of the Total Environment*.

[4] Darby S. C., Whitely E., Howe G. R. (1995). Radon and cancers other than lung cancer in underground miners: a collaborative analysis of 11 studies. *Journal of the National Cancer Institute*.

[5] Turner M. C., Krewski D., Chen Y., Pope C. A., Gapstur S. M., Thun M. J. (2012). Radon and COPD mortality in the American cancer society cohort. *European Respiratory Journal*.

[6] Kreuzer M., Grosche B., Schnelzer M., Tschense A., Dufey F., Walsh L. (2010). Radon and risk of death from cancer and cardiovascular diseases in the German uranium miner’s cohort study: follow-up 1946–2003. *Radiation and Environmental Biophysics*.

[7] Morrison H. I., Semenciw R. M., Mao Y., Wigle D. T. (1988). Cancer mortality among a group of fluorspar miners exposed to radon progeny. *American Journal of Epidemiology*.

[8] Navaranjan G., Berriault C., Do M., Villeneuve P. J., Demers P. A. (2016). Cancer incidence and mortality from exposure to radon progeny among Ontario uranium miners. *Occupational and Environmental Medicine*.

[9] Darby S., Hill D., Auvinen A. (2005). Radon in homes and risk of lung cancer: collaborative analysis of individual data from 13 European case-control studies. *BMJ*.

[10] Radon and Public Health (2009). Report of an independent advisory group on ionising radiation. *Chilton, Docs RCE*.

[11] Tirmarche M., Harrison J. D., Laurier D. (2010). ICRP Publication 115. Lung cancer risk from radon and progeny and statement on radon. *Annals of the ICRP*.

[12] http://apps./who.int/gho/data/view.main.

[13] Henschel Invited D. (1994). Analysis of radon mitigation techniques used in existing US houses. *Radiation Protection Dosimetry*.

The article "Assessment of Seasonal Radon Concentration in Dwellings and Soils in Selected Areas in Ga East, Greater Accra Region of Ghana" was published in 2022. Journal: J Environ Public Health.

[14] Cosma C., Papp B., Cucoş Dinu A., Sainz C. (2015). Testing radon mitigation techniques in a pilot house from Băiţa-Ştei radon prone area (Romania). *Journal of Environmental Radioactivity*.

[15] Leovic K. W., Sanchez D. C., Craig A. B. (1988). Radon mitigation choices in the United States-a comparison of private and public sector developments. *Radiation Protection Dosimetry*.

[16] World Health Organization (2009). *WHO Handbook on Indoor Radon: A Public Health Perspective*.

[17] Nsiah-Akoto I., Fletcher J. J., Oppon O. C., Andam A. B. (2011). Indoor radon levels and the associated effective dose rate determination at Dome in the Greater Accra Region of Ghana. *Research Journal of Environmental and Earth Sciences*.

[18] Oppon O. C., Aniagyei H. M., Kyere A. W. K. (1993). Monitoring of natural Background radiation in some Ghanaian homes. *High levels of natural radiation*.

[19] Quashie F. K. (2010). *Indoor Radon Measurement in Some Adobe Houses in the Kassena Nankana Area of the Upper East Region*.

[20] Andam A. A. B. (1994). Radon levels in sub-soil and local building materials. *Journal of Radiological Protection*.

[21] Amponsah P., Banoeng -Yakubo B., Andam A., Asiedu D. (2008). Soil radon concentration along fault systems in parts of south eastern Ghana. *Journal of African Earth Sciences*.

[22] Kesse G. O. (1985). *The Mineral and Rock Resources of Ghana*.

[23] Laux P., Kunstmann H., Bárdossy A. (2008). Predicting the regional onset of the rainy season in West Africa. *International Journal of Climatology*.

[24] Kitson-Mills D., Sovoe S., Opoku-Ntim I. (2019). An assessment of indoor radon level in a suburb of Ghana. *Environmental Research Communications*.

[25] Bhagwat A. M. (1993). *Solid State Nuclear Track Detection: Theory And Applications (No. ISRP-K-TD--2)*.

[26] Yu K. N., Nikezic D., Ng F. M. F., Leung J. K. C. (2005). Long-term measurements of radon progeny concentrations with solid-state nuclear track detectors. *Radiation Measurements*.

[27] Nsiah-Akoto I. (2017). Radon—occurrence, risk estimation, and mapping of levels in the water, indoors, and soil in obuasi and offinso in the ashanti region.

[28] Omar A. S. (2020). Radium content and radon exhalation rates in Egyptian soil samples using active and passive techniques. *Radiation Protection and Environment*.

[29] Amponsah P. E., Andam A. B., Nsiah-Akoto I. (2015). Radon measurements in soils along the coast of Accra from teshie to nyanyano, southeastern Ghana. *Environmental Research, Engineering and Management*.

[30] ICRP publication 65 (1993). International commission on radiological protection. Protection against radon-222 at home and work. *Annals of the ICRP*.

The article "Assessment of Seasonal Radon Concentration in Dwellings and Soils in Selected Areas in Ga East, Greater Accra Region of Ghana" was published in 2022. Journal: J Environ Public Health.

[31] Collignan B., Le Ponner E., Mandin C. (2016). Relationships between indoor radon concentrations, thermal retrofit, and dwelling characteristics. *Journal of Environmental Radioactivity*.

[32] Ajayi O. S., Olubi O. E. (2016). Investigation of indoor radon levels in some dwellings of southwestern Nigeria. *Environmental Forensics*.

[33] Çelik N., Çevik U., Çelik A., Kucukomeroglu B. (2008). Determination of indoor radon and soil radioactivity levels in Giresun, Turkey. *Journal of Environmental Radioactivity*.

[34] Chege M. W., Rathore I. V. S., Chhabra S. C., Mustapha A. O. (2009). The influence of meteorological parameters on indoor radon in selected traditional Kenyan dwellings. *Journal of Radiological Protection*.

[35] Hámori K., Tóth E., Pál L., Köteles G., Losonci A., Minda M. (2006). Evaluation of indoor radon measurements in Hungary. *Journal of Environmental Radioactivity*.

[36] Khan F., Ali N., Khan E. U. (2012). Study of indoor radon concentrations and associated health risks in the five districts of Hazara division, Pakistan. *Journal of Environmental Monitoring*.

[37] Farid S. M. (2016). Indoor radon in dwellings of Jeddah city, Saudi Arabia and its correlations with the radium and radon exhalation rates from soil. *Indoor and Built Environment*.

[38] Nsiah-Akoto I., Andam A. B., Akiti T. T., Flectcher J. J., Osei P. Indoor radon mapping: the Ghanaian strategy.

[39] Stojanovska Z., Januseski J., Bossew P., Zunic Z. S., Tollefsen T., Ristova M. (2011). Seasonal indoor radon concentration in FYR of Macedonia. *Radiation Measurements*.

[40] Miles J. C. H., Howarth C. B., Hunter N. (2012). Seasonal variation of radon concentrations in UK homes. *Journal of Radiological Protection*.

[41] Karpińska M., Mnich Z., Kapała J. (2004). Seasonal changes in radon concentrations in buildings in the region of northeastern Poland. *Journal of Environmental Radioactivity*.

[42] Chen J., Ford K. L. (2017). A study on the correlation between soil radon potential and average indoor radon potential in Canadian cities. *Journal of Environmental Radioactivity*.

[43] King C. Y., Minissale A. (1994). Seasonal variability of soil-gas radon concentration in central California. *Radiation Measurements*.

[44] Winkler R., Ruckerbauer F., Bunzl K. (2001). Radon concentration in soil gas: a comparison of the variability resulting from different methods, spatial heterogeneity, and seasonal fluctuations. *Science of the Total Environment*.

[45] Moreno V., Bach J., Font L. (2016). Soil radon dynamics in the Amer fault zone: an example of very high seasonal variations. *Journal of Environmental Radioactivity*.

